# Alcohol consumption and hormonal alterations related to muscle hypertrophy: a review

This article has been retracted.

**DOI:** 10.1186/1743-7075-11-26

**Published:** 2014-06-06

**Authors:** Antonino Bianco, Ewan Thomas, Francesco Pomara, Garden Tabacchi, Bettina Karsten, Antonio Paoli, Antonio Palma

**Affiliations:** 1 Sport and Exercise Sciences Research Unit, University of Palermo, Via Eleonora Duse, 2, 90146 Palermo, Italy; 2 MEDEOR Research Institute, Via Emilio Salgari, 69, 90147 Palermo, Italy; 3 Department of Sciences for Health Promotion and Mother-Child Care “G. D’Alessandro”, University of Palermo, Via del Vespro 133, 90127 Palermo, Italy; 4 Life and Sports Science, University of Greenwich, Central Avenue, ME4 4TB, Chatham Maritime, United Kingdom; 5 Department of Biomedical Sciences (DSB), University of Padova, Via Marzolo 3, 35131 Padova, Italy

**Keywords:** Alcohol, Muscle hypertrophy, Hormones, Protein synthesis

## Abstract

Detrimental effects of acute and chronic alcohol (ethanol) consumption on human physiology are well documented in the literature. These adversely influence neural, metabolic, cardiovascular, and thermoregulatory functions. However, the side effects of ethanol consumption on hormonal fluctuations and subsequent related skeletal muscle alterations have received less attention and as such are not entirely understood. The focus of this review is to identify the side effects of ethanol consumption on the major hormones related to muscle metabolism and clarify how the hormonal profiles are altered by such consumption.

## Introduction

Hormones are chemical messengers that control and coordinate the functions of all tissues and organs [1]. Each hormone is secreted from a particular gland and distributed throughout the body to act on tissues at different sites. Two areas of the brain, the hypothalamus and the pituitary, release hormones, as do glands in other parts of the body [2]. Hormones control four major areas of body function: production, use, and storage of energy; reproduction; maintenance of the internal environment; and growth and development [3-6]. For hormones to function properly, their amount and the timing of their release must be finely coordinated, and the target tissues must be able to respond to them accurately. Ethanol can impair the functions of the hormone-releasing glands and of the target tissues, thereby causing medical consequences [7].

Nowadays alcohol consumption in western countries is considerably increasing [8-10] and it is common knowledge, that acute, regular or excessive ethanol consumption has detrimental effects on human physiology. For example, ethanol ingestion affects many aspects of metabolism as it impairs hepatic gluconeogenesis and subsequent glucose output and storage [11,12].

It is also well documented that glucose availability is used to fuel muscle protein synthesis during recovery from exercise [13]; these conditions highlight how ethanol ingestion could have negative consequences for muscle metabolism.

Furthermore, ethanol causes an increase in adrenal gland secretion of steroid hormones, which stimulates the anterior pituitary gland to secrete the Adrenocorticotropic hormone (ACTH) [14-16]. ACTH acts on the cortical zone of the adrenal gland and stimulates the formation of mineral corticoids, in particular of aldosterone and glucocorticoids. Both mineral corticoids affect the metabolism of sugars and androgens which in turn affect the metabolism of skeletal muscle [17,18]. Acute alcohol consumption also impacts on neural function, cardiovascular function, thermoregulatory function and can cause skeletal muscle myopathyes such as the alcoholic myopathy [19-21].

The understanding of hormone variations as a consequence of alcohol consumption is fundamental to understand how muscle hypertrophy could get impaired. This review aims to provide an insight into current knowledge of the interactions between alcohol consumption and the related hormonal alterations that could alter muscle hypertrophy.

## Review

### Methods

We manually researched studies through PUBMED, SCIRUS and SCIENCE DIRECT from 1975 to 2013 and all citations inserted through EndNote X6 ©1988-2012 Thomson Reuters. The search included studies that related ethanol consumption to: skeletal muscle, sport, hypertrophy, hormones and overall physiological alterations. Our research produced 106 results. All information was consequently divided in two major categories: 1) “Muscle hypertrophy mechanisms” where we tried to elucidate the different biological mechanisms involved in muscle hypertrophy to subsequently understand how ethanol impacts on these mechanisms and 2) “Alcohol and hormonal alterations” in which the relationship between ethanol consumption and different hormonal profiles linked to muscle metabolism are clarified.

#### Muscle hypertrophy mechanisms

Generally there are two mechanisms for which proteins may accumulate during growth or training and thus induce hypertrophy: the first is an increase in protein synthesis and the second is a reduction in the rate of degradation [22,23]. In adults, muscle proteins are constantly being replaced with a turnover of about 7–15 days. The final balance between anabolism and catabolism is the expression of the relationship between protein synthesis and degradation [24,25]. It seems there is no difference in the rate of protein turnover between different muscle fibre types [26] but we also know that fast twitch muscle fibres are more responsive to hypertrophy [27,28]. Exercise aimed at increasing muscle mass is associated with changes in one or more of the following variables: muscle passive tension; contraction induced tension; sarcoplasmatic calcium concentration; energy demand; intramuscular oxygen concentration; hormonal presence; growth factors and cytokines; temperature and cell damage [29-31]. A sufficient change in one of these variables can lead to an alteration in the activity of signal transduction pathways that regulate the transcription of genes involved in muscle growth [31,32].

The most important pathways are those which involve proteins with kinase or phosphatase activity and molecules which catalyze the addition or removal of a phosphate group to, or from a specific substrate [33-36]. Exercise, at any given time, activates more than one of these pathways, which indicates that the muscle hypertrophy phenomenon is complex and multifactorial. One of the main mechanism that regulates protein synthesis involves ribosomal protein translation with transcription of messenger ribonucleic acid (mRNA) [37-39].

In addition, the activation of protein kinase mechanistic target of rapamycin (mTOR) is implicated in the control of protein synthesis. Once activated, mTOR phosphorylates specific proteins that phosphorylate and activate another protein kinase termed ribosomal protein S6 kinase (S6K). The S6K triggers a cascade of responses that subsequently phosphorylate ribosomal protein S6 [40].

Phosphorylation of the specific eukaryotic translation initiation factor 4E (eIF4E) promotes the initiation of a series of mRNA rapid translation which encodes proteins necessary for protein synthesis. This pathway is activated during physical activity [41,42] and appears to be responsible for the increase in slow twitch fibres proportion [43,44]. The activation of S6K and mTOR is essential for muscle hypertrophy and is associated with the signal that arrives at the PKB/AKT pathway by Phosphoinositide 3-kinase (PI3) in vivo where the insulin like growth factor 1 (IGF-1) also appears to act [42]. Figure 1 shows where ethanol is implicated in the inhibition of protein synthesis.

**Figure 1:** **Molecular interactions between EtOH and IGF-1.** Metabolic pathways and signals of IGF-1: The schematic representation emphasizes the primary role of the cascade PI(3)K/Akt [25]. The figure also shows where alcohol impairs muscle hypertrophy mechanisms.

Other hypertrophy mechanisms are hormonally related. Testosterone and the growth hormone (GH) are the two main anabolic hormones. The first with anabolic effects on protein synthesis by acting directly at a nuclear level. The latter has an anabolic effects by acting through another growth factor: the IGF-1. This is considered as a possible mediator in the action of overload. Indeed, through the release of IGF-1, local overload applied to a muscle induces an increase in muscle mass, stimulating PI3 kinase and Akt [45]. Moreover, IGF-1 alone can stimulate hypertrophy [45].

### Protein synthesis and alcohol consumption

Ethanol and its metabolic secondary products, such as acetaldehyde directly affect protein synthesis in skeletal muscle tissue [46-48]. Main affected muscle fibres are type II, especially type IIx [49,50]. It is known that type IIx fibers are those more responsive to hypertrophy [51]. A decrease in basal protein synthesis by 15% to 20% was observed in skeletal muscle after 24 hr of ethanol intoxication [52].

Incubation of myocytes for 72 hr decreased synthesis in cells incubated with ethanol (EtOH) ranging between 60 and 120 mM. The ability of IGF-I or insulin to stimulate protein synthesis was impaired by 30% and 60%, respectively, in cells incubated with 80 mM of ethanol for 72 hr. It has to be noted though, that such concentrations (60 and 120 mM) would correspond in vivo to a blood alcohol content (BAC) of 0.276% and 0.55%, respectively. Moreover, exposure of cells to 200 μM acetaldehyde or 5 mM Na-acetate also decreased basal protein synthesis. In contrast, neither ethanol, acetaldehyde nor acetate altered the basal rate of protein degradation.

Although, ethanol compromised the ability of both insulin and IGF-I to slow proteolysis [52]. Furthermore, ethanol consumption may suppress protein synthesis slightly via inhibition of exercise-induced mTOR, which is partially dependent on phosphatidic acid (PA) from the cell membrane for complex stabilization [53]. Ethanol is used as preferential substrate by the enzyme Phospholipase D and phosphatidylethanol is produced in lieu of PA, which causes an indirect suppression of mTOR [54]. It appears to act more on the mTORc1 subcomponent, as higher concentrations are needed to inhibit the mTORc2 component [53,54]. This mechanism of action has been demonstrated acutely with mouse myocytes [55] and chronic alcoholism adversely affects mTOR and S6K1 phosphorylation [56,57]. Ethanol so selectively impairs IGF-I signalling via S6K1, but not Eukaryotic translation initiation factor 4E binding protein 1 (4E-BP1), and this is independent of gender, nutritional state, route of administration, and ethanol metabolism. Experimental studies also suggest that myocyte myostatin increases with ethanol exposure [58]. Myostatin is the growth differentiation factor-8 (GF-1b), a potent inhibitor of skeletal muscle and heart growth [59]. Myostatin controls cell cycle progression and inhibits skeletal myoblast proliferation and terminal differentiation. An increase in myostatin activity protects the cell from apoptosis. Its disruption causes increased skeletal mass with hypertrophy and hyperplasia of myocytes and increased myocyte proliferation [60]. The outcomes of the study of Lang et. al indicate that chronic alcohol feeding for 16 wk increases the myostatin mRNA content in the gastrocnemius. Moreover, 3-day treatment of alcohol-fed rats with IGF-I/IGFBP-3 reversed the increase in muscle myostatin mRNA. Constitutive expression of myostatin mRNA in muscle from control rats was relatively low. Although the basal and IGF-I-induced changes in myostatin mRNA are consistent with the observed changes in muscle protein mass determined in alcohol-fed rats [58]. IGF-I resistance may represent a participating mechanism by which ethanol directly limits the translation of selected messenger RNAs and ultimately protein synthesis in skeletal muscle [61]. Ethanol did not impair IGF-I receptor autophosphorylation, but inhibited the ability of insulin to phosphorylate its own receptor. Ethanol also did not alter the number of insulin or IGF-I receptors or the formation of insulin/IGF-I hybrid receptors [52,61] that added to the hormonal imbalance above mentioned can lead to atrophy [31,47,62].

Moreover another study measuring liver protein kinetics has found that in humans pairing a meal of 632 kcal with ethanol (71 g), reduced the protein synthesis rate (assessed by fibrinogen and albumin) by about 30% over the 4 hours measured afterwards; this study also noted that leucine oxidation (a marker of muscle protein breakdown) was reduced by 24% [63]; it was also found, using labelled leucine to measure the fractional secretory rate of hepatic proteins, that a moderate dose of alcohol (28 g, approximately 2 drinks) slightly affect postprandial hepatic protein metabolism by blunting the meal-induced increase in albumin synthesis [64]. A subsequent study confirmed that ethanol, compared to saline control, was able to suppress leucine oxidation at two varying doses and this apparent anti-catabolic action was more effective when no circulating nutrients were present [65].

#### Alcohol and hormonal alterations

As described a multitude of mechanisms which regulate muscle hypertrophy are hormone mediated. Indeed the hormonal profile is fundamental in determining whether the outcome is protein synthesis or protein degration. Knowledge of the effects of ethanol consumption on these mechanisms will provide a clearer view about the relationship between skeletal muscle hypertrophy and alcohol.

### Testosterone

Moderate doses of ethanol (0.83 g/kg) in resistance trained men when consumed immediately after exercise (where nothing was eaten 3.5 hours before, food given during drinking ab libitum) failed to note any significant differences in testosterone levels for up to 300 minutes after exercise [66] and another sport related study using 1 g/kg after a simulated rugby match failed to note a decrease in testosterone despite noting a reduction in power output [67]. Rojdmark et al. did not pair ethanol with exercise but used a low dose of 0.45 g/kg on three separate pulses. 90 minutes apart noted that although there was a trend for testosterone to increase that did not differ between ethanol and water intake [68]. Conversely, a slightly lower intake (0.5 g/kg) has been shown to actually increase circulating testosterone from 13.6 nmol/L to 16 nmol/L (+17%) 2 hours after ingestion [69]. This increase in testosterone after 0.5 g/kg has also been noted in premenopausal women [70] and suggested to act vicariously through the increased NADH/NAD + ratio in the liver after these doses. Steroid metabolism and REDOX couplets interact in the liver [71], where an increased rate of 17β-Hydroxysteroid dehydrogenases (17β-HSD) type 2 enzyme and its conversion of Androstenedione (ASD) to testosterone is observed due to the increased NADH relative to NAD + observed after ethanol intake, and this also explains the reduction in ASD observed in studies where testosterone is increased [70,71] and may help explain the increased levels of ASD in studies where testosterone is suppressed, where ASD may be increased by up to 54% (and DHEA by 174%) 12 hours after large intakes of ethanol [72]. That being said, another study using 0.675 g/kg of ethanol noted that testosterone increased and was more sensitive to being increased by gonadotropin releasing hormone, suggesting multiple pathways may be at play [73]. Red Wine may also confer additional benefits through its phenolic content, as Quercetin (A plant-derived antioxidant flavonoid found in red wine, green tea, onions, apples and leaf vegetables [74]. It has been reported that decreases oxidative DNA damage induced by reactive oxygen species, such as H2O2 and tert-butylhydroperoxide. Thus, dietary consumption of quercetin can reduce the risk of multiple diseases associated with oxidative stress [75]. It has been also been reported to possess unique anti-apoptotic proprieties in male germ cells [76]) appears to be glucuronidated by the enzyme UGT2B17 in place of testosterone (sacrificial substrate) and may indirectly increase testosterone [77]. Though, this study was in vitro and Quercetin has low bioavailability.

Higher doses of ethanol, 1.5 g/kg (average dose of 120 g), have been demonstrated to suppress testosterone by 23% when measured between 10–16 hours after acute ingestion with no statistical significant difference between 3 and 9 hours of measurement. It appeared that ethanol suppressed a rise of testosterone that occurred in the control group which may have been based on the circadian rhythm [78]. Another study using higher dosages (1.75 g/kg over 3 hours) noted that after 48 hours a small short-lived dip occurred, but a higher statistically significant drop was seen at 12 hours which was mostly corrected after 24 hours from ingestion (still significantly less than control) and completely normalized at 36 hours. By 12 hours, the overall reduction in testosterone was measured at 27% while the overall decrease in testosterone at 24 hours was 16% [72]. A third study using vodka at a dose of 2.4 ml/kg bodyweight in 15 minutes (to spike BAC up to 109+/−4.5 mg/100 mL, similar to the aforementioned 1.75 g/kg study) noted suppressed testosterone levels correlating with the BAC peak, observed 84 minutes after ingestion [79]. This time delay seen in some studies, when put in social context, correlates with the observed lower serum testosterone levels seen with hangovers [80]. Finally, an intervention in which ethanol was supplied intravenously (via catheter) to keep a breath ethanol level of 50 mg%, noted that free testosterone was suppressed at this level of intake in young (23+/−1) men only, with young women experiencing an increase in testosterone and older (59+/−1) men and women having no significant influences [81]. Around the 1.5 g/kg or higher ethanol intake, it appears that a dose-dependent decrease of testosterone occurs and appears to occur with some degree of time delay up to 10 hours after consumption. However, the acute intake of ethanol of about 1.5 g/kg suppresses the production of testosterone within one hour through a decrease in Luteinizing hormone (LH) release [82]. The study of Cicero et al. used shots of vodka and noted this suppression of testosterone occurring within 90 minutes though. In ethanol abusers, the chronic high intake of ethanol appears to be negatively correlated with circulating testosterone at rest; with longer duration and higher intakes of ethanol leading to less testosterone [83]. As suggested by Heikkonen and Barnes [67,84] the decreased testosterone levels might have been due to differences in ethanol administration (dosage/timing).

Hormonal levels of testosterone have also been measured after heavy resistance exercise [85]. Participants consumed either 1.09 g/kg of grain ethanol per kilogram lean mass (EtOH group) or no ethanol post exercise (placebo group). Peak blood ethanol concentration (0.09 ± 0.02 g · dL) was reached within 60–90 min post exercise. Total testosterone and free testosterone were elevated significantly immediately after exercise in both groups. At 140–300 min post exercise, total testosterone and free testosterone levels as well as free androgen index were significantly higher only in the EtOH group. The study demonstrated that during the recovery period from heavy resistance exercise, post exercise ethanol ingestion affects the hormonal profile including testosterone concentrations and bioavailability [85].

A number of studies have highlighted the decrease in testosterone levels after ethanol consumption by synthesis inhibition and release of testosterone by the testes [13,14,84,86]. The mechanism of ethanol suppressing testosterone levels sub-chronically is via its actions as a testicular toxin, where it can reduce testosterone synthesis rates with no negative influence on the hypothalamus signals to the testes [83,87]. Ethanol locks the functionality of Leydig cells [88] and it has been shown that necrotic Leydig cells were evident after chronic ethanol consumption [88-90]. Although, in females, the production and release of androgens occurs outside the gonads. Therfore the action of ethanol on LH levels on Leydig cells is irrelevant. Testosterone production occurs in the adrenal glands as an intermediate in the synthesis of cortisol. Ethanol stimulates adrenal gland activity [91] and increased levels of ethanol consequently results in an increase in androgen hormones in females [92,93].

### Main findings

There appears to be a dose dependency in the hormonal response. All the studies that analyzed testosterone using a dose lower than 1.5 g/kg show an increase in the circulating levels of the hormone. Conversely all those using higher dosages (1.5 g/kg ) show a decrease. It also seems that the decrease can only be seen in men while an increase is evident in women.

### Estrogen

A three week intervention in middle aged men and post-menopausal women drinking 30-40 g of alcohol daily noted that in both genders there was no significant influence of this dose of ethanol on circulating estrogen levels [94].

Another study measuring serum levels during hangover (induced by 1.5 g/kg ethanol the night prior) noted less circulating estrogen levels associated with hangover [80] yet another study using similarly high levels of 1.75 g/kg ethanol noted no significant influence of ethanol on estrogens for the next 48 hours measured, if anything a slight trend to decrease estrogens was noted [72].

There is a strong possibility though that ethanol increases the aromatization of androgens [95]. Ginsburg and collegues have shown that ethanol consumption can increase estradiol levels by up to 300% [96] as changes in hepatic redox states associated with the catabolism of ethanol [96] and so lead to hormonal imbalances with further decreases in anabolic hormones [97,98].

### Main findings

Two studies show no difference between estrogen levels before and after alcohol consumption. Although at higher doses than those used in the previous mentioned studies contradictive results show an increase in women and a decrease in men.

### Cortisol

After consumption of 1.75 g/kg ethanol, a spike in cortisol is seen at 4 hours and persists for up to 24 hours after consumption, normalizing at 36 hours [72]. At 4 hours, the greatest spike of cortisol seen, was measured to be 152% higher than control and this increase in cortisol does not appear to correlate to the decrease in testosterone as shown in Figure 2[72,99].

**Figure 2:** **Plasma cortisol concentrations after EtHO ingestion.** Plasma cortisol concentrations measured from the beginning of the infusion period every 30 minutes for 2 to 24 hours. The infusion of 1.75 g/kg of ethanol significantly increased maternal plasma cortisol concentrations at 1, 1.5 and 2 hours compared to all other treatment groups. Reprint with permission by Ramadoss et al. [99].

Ethanol furthermore increases the level of cortisol through the release of ACTH [15,100,101]. Murphy et al. [102] analyzed the influence of ethanol consumption during competitive rugby league matches recovery. The researchers found a significant increase in cortisol levels with no changes in the level of testosterone [102].

### Main findings

Studies show an increase in the level of cortisol. It is not clear if this increase is due to the stress that the organism undergoes as a consequence of alcoholic ingestion or to an increase in the level of ACTH.

### Growth and Luteinizing hormones

Physiological and sport induced alterations are well documented in the literature regarding GH and LH [103,104], but little is known about their kinetics after ethanol consumption. Ylikahri et al. [105] found that ethanol had no significant effects on basal concentrations of GH after administration of a large dose of ethanol (1.5 g/kg BW). Contrary to Ylikahri, Tentler et al. [106] identified that ethanol caused prolonged and severe decrease in serum GH, possibly mediated at secretion level. Another study indicates that GH does not appear to have its pulse amplitude influenced by ethanol for up to 20 hours after ingestion of a large dose (1.5 g/kg) of ethanol acutely in otherwise healthy men. However, pulse frequency during these 20 hours was slightly but significantly reduced (from 4.7+/−0.2 to 3.8+/−0.3) [78].

Ethanol inhibits the release of the gonadotropin-releasing hormone (GnRH) at an hypothalamic level. With a signaling role on the pituitary gland of GnRH to release LH, an increase in BAC consequently leads to a decrease in LH levels which in turn partially results in lower testosterone production in adults and adolescents [13,84,100,101].

### Main findings

The GH shows a serum level decrease in four out of five analyzed the studies. No alterations were shown in the remaining study. Whereas for the LH a decrease was shown in all analyzed studies.

## Conclusions

Research results confirm the detrimental effects of ethanol ingestion on a multitude of physiological levels. Protein synthesis and resulting muscle hypertrophy appears to be directly affected by ethanol. Ethanol and its metabolic sub-products selectively impair IGF-I signalling via S6K1 that directly affects the transcription of genes involved in muscle hypertrophy especially in type IIx fibers, those more responsive to hypertrophy. A direct link between ethanol consumption and hormonal profiles is evident. These links indicate that ethanol reduces GH plasmatic levels and alters the pituitary axes by decreasing LH release, which consequently, depending on the dose consumed could induce a decrease in the level of testosterone. Furthermore ethanol and its metabolic sub-products, inhibit testosterone but also increases cortisol levels, an opposite trend on muscle hypertrophy achievement. Though, the findings seem to be contradictive; the role of ethanol on cortisol and testosterone secretion is still not entirely understood but the stressful effects of ethanol onto the human body may be responsible for the increase in cortisol serum levels in a number of studies. Moreover, alterations in testosterone levels appear to be gender specific. A decrease in secreted testosterone has been shown in males whilst an increase due to the activation of the adrenal axes has been shown in females.

Interestingly in 100% of analysed studies, an ethanol dose administration greater than 1.5 g/kg showed a decrease in testosterone serum levels. This underlines a dose dependent physiological mechanism related to ethanol consumption (Assuming that a glass of beer is around 12 oz (355 ml) and on average it’s alcohol content is between 4.5 and 6%, for a 70 Kg man this dose would correspond to 5–6 glasses of beer). No differences between adolescents and adults were identified.

If a reduced level of blood testosterone is present, a reduced protein synthesis should occur in males and this would lead to atrophy.

This review has identified a lack of information about the specific and direct interaction between ethanol and muscle hypertrophy. Furthermore, the majority of studies related to the topic are often dated with conflicting results being evident. Ethical considerations to ethanol consumption and/or intoxication in *in vivo* studies might be the cause of low publication numbers. This study underlines to scientist involved in the field of exercise nutrition the need to inform athletes and sport professionals on the possible effects and implications that the consumption of this substance could cause.

## Abbreviations

4E-BP1: Eukaryotic translation initiation factor 4E binding protein 1; 17β-HSD: 17β-Hydroxysteroid dehydrogenases; ACTH: Adrenocorticotropic hormone; Akt: Protein Kinase B; ASD: Androstenedione; DHEA: Dehydroepiandrosterone; EtHO: Ethanol; eIF4E: Eukaryotic translation initiation factor 4E; GH: Growth Hormone; GnRH: Gonadotropin-releasing hormone; IGF-1: Insulin-like growth factor 1; mRNA: Messenger Ribonucleic acid; mTOR: Mechanistic target of rapamycin; NAD^+^/NADH: Nicotinamide adenine dinucleotide; PA: Phosphatidic acid; Pi3: Phosphoinositide 3-kinase; S6K: Ribosomal protein S6 kinase.

## Competing interests

The authors declare that they have no competing interests.

## Authors’ contributions

AB, ET and AP conceived and designed the manuscript. FP, GT, BK critically reviewed the manuscript drafts. AB, ET, AP and APal drafted the manuscript. All authors read and approved the final manuscript.
